# Sensing risk, fearing uncertainty: systems science approach to change

This article has been retracted.

**DOI:** 10.3389/fncom.2014.00030

**Published:** 2014-03-31

**Authors:** Ivo P. Janecka

**Affiliations:** Foundation for Systems Research and EducationNew York, NY, USA

**Keywords:** change, risk, uncertainty, systems science, chaos, entropy, cancer, neuro-degeneration

## Abstract

**Background:** Medicine devotes its primary focus to understanding *change*, from cells to network relationships; observations of non-linearity are inescapable. Recent events provide extraordinary examples of major non-linear surprises within the societal system: *human genome*-from anticipated 100,000+ genes to only 20,000+; *junk DNA*-initially ignored but now proven to control genetic processes; *economic reversals*-bursting of bubbles in technology, housing, finance; *foreign wars*; relentless *rise in obesity, neurodegenerative diseases.* There are two attributes of systems science that are especially relevant to this research: One—it offers a method for creating a structural context with a guiding path to pragmatic knowledge; and, two—it gives pre-eminence to sensory input capable to register, evaluate, and react to *change*.

**Materials/Methods:** Public domain records of *change*, during the last 50 years, have been studied in the context of systems science, the dynamic systems model, and various cycles.

**Results/Conclusions:** *Change* is dynamic, ever-present, never isolated, and of variable impact; it reflects innumerable relationships among contextual systems; *change* can be perceived as risk or uncertainty depending upon how the assessment is made; risk is quantifiable by sensory input and generates a degree of rational optimism; uncertainty is not quantifiable and evokes fear; trust is key to sharing risk; the measurable financial credit can be a proxy for societal trust; expanding credit dilutes trust; when a credit bubble bursts, so will trust; absence of trust paralyzes systems' relationships leading to disorganized complexity which prevents value creation and heightens the probability of random events; disappearance of value, accompanied by chaos, threatens all systems. From personal health to economic sustainability and collective rationality, most examined components of the societal system were found not to be optimized and trust was not in evidence.

## Introduction

Surprising developments, sudden reversals, and major upheavals have been part of human experience since the beginning of recorded history and can be broadly categorized as *change*. Any new *change* disturbs the dynamic richness of the existing environment and its inter-related systems; through forms of interference, it leaves its imprint. Harnessing senses and cognition, a biologic system can unlock enough of the imprint's pattern of *change* for critical comprehension.

*Change* is an alteration of a previous state of existing relationships. The dominant link between *change* and systems science is the foundational premise that everything is, in some way, connected to everything else, implying a broad interconnectedness of all open systems. Any *change* can alter the spectrum of upstream as well as downstream relationships. The ability to adapt and evolve with *change* are prerequisites for any successful system; both features are expressed in a dynamic construct of integration, relevancy, and accountability generated from sensory input of data, processed information, and the created knowledge.

The purpose of this study is to make *change* more manageable; the path, to reach this goal, is to differentiate it into what is potentially quantifiable and what is not. Risk, as defined in this study and with applicability to human bodily system, is considered quantifiable through sensory input which also generates a degree of experiential confidence and predominantly rational optimism; what is outside of sensory spectrum is regarded as unquantifiable uncertainty which evokes emotions such as fear, greed, irrationality, etc. The advantage of separating sensory-defined risk from the remaining uncertainty is that it isolates a portion of *change* whose outcome has a relatively high degree of predictability; uncertainty has none as it has random outcome.

To improve the odds of understanding and pragmatically coping with *change*, is to convert as much of existing uncertainty into quantifiable risk by employing relevant primary and, when feasible, technology-expanded sensory processing. For example, a microscope, a telescope, a night vision scope, surgical navigation, etc. can be used to magnify and refine our vision; sensitive amplifiers can augment our auditory processing, etc. The specific senses that are used, however, need to be highly appropriate for the character of the *change* under study with the comprehension that each sense has a range and detection limitations expressed as sensitivity and specificity; risk-uncertainty (R/U) ration can be created but how the ratio is constructed and how its impact is judged, however, varies greatly. The R/U ration, from an identical *change*, may vary significantly in its influence across differing living systems based on their own capacity to create organized complexity and value/emergence—essentially, expressions of state of health of their systems.

A full comprehension of any *change*, its real-life R/U ration, depends on the contextual understanding of both the system that generates the *change* and all other systems that are in its path. System science offers valuable understanding of *change* that reverberates through systems' inter-relationships. *Change*, therefore, is not an isolated event, and, depending upon compliance of the engaged systems with the principles of systems science, the impact of *change* can range from a minor “ripple” to a major “Tsunami.”

Systems science has been selected as the primary research tool as it offers a comprehensive perspective and a framework for evaluating multidimensionality of *change* as well as offering a range of likely outcomes. Some systems science principles are more visible on different levels of biologic systems, extending from cellular to societal level. To best illustrate some of the key points, examples from such various systems have been selected; some terms/concepts of systems science represent a compressed coil of meanings; for better understanding, metaphors are being used.

This research is based on observations of others, as I understand them, as well as my own. Biologic principles, as systems science tries to emulate, are, as biology itself, still incompletely understood and always *changing*, epitomizing the essence of *change* itself. Any observed principles are only transient, even if the transition spans a very long time. None the less, there is an endless learning in the subject as we are just a part of the same biology that we study.

Though von Bertalanffy is credited with recent (1960s) focus on systems science arising from observations of biologic principles, search of history can be revealing. For example, Lao-Tzu (cca sixth century BC) taught, in ancient China, the importance of awareness of self as being part of the overall Nature; systems science would categorize it as a view of all-systems inter-relatedness. Later, Confucius (551–479 BC) focused his teachings on the need for relationships to be based on fairness and trust as the hallmarks of morality; systems science perspective expresses that optimizing relationships need to be reciprocal, fair, empathic, and based on trust (von Bertalanffy, 1969; Laozi, 1900; Ames and Rosemount Jr, 1999).

The prevailing thesis of this research progresses along the following conceptual outlines:

- *Change* is dynamic, ever-present, never isolated, and of variable impact; it reflects innumerable relationships among contextual systems, from individuals to a society; *change* can be perceived primarily as risk or uncertainty depending upon how and by whom the assessment is made; risk is quantifiable by sensory input and generates a degree of rational optimism; uncertainty is not quantifiable by this path and evokes fear; trust is key to sharing risk, maintaining social bonds, and optimizing a societal system; the quality/quantity of measurable financial credit can be an inverse proxy for the level of societal trust as expanding credit dilutes trust; the absence of trust negatively impacts system's relationships leading to disorganized complexity which prevents value creation and heightens the probability and severity of random events; when a credit bubble busts, so does trust; any further over-expansion of credit fails to stimulate the economy which represents socioeconomic relationships; disappearance of value, concomitantly with trust, threatens the entire system, which is considered to be in chaos; the fundamental corrective steps must focus on the re-establishment of trust.
- Recent events have provided extraordinary examples of major and unanticipated *changes* within the societal system for which definite answers are still pending. For example, the human genome was anticipated to have 100,000+ genes, in order to satisfy the linear extrapolation of a concept, schematically expressed as: one disease-one gene. But, only 20,000+ genes were actually found; 10,000+ fewer than a tomato or little clump of moss. The difference, in number of genes that favors non-human organisms and the vast functionality of human beings, likely lies in the non-linear ability of genes for alternate splicing: individual genes are UP/DOWN regulated, combined and re-combined in fractal, non-linear patterns serving an array of functions.

### Anticipated obstacles to the implementation of this research

Persistent belief in linearity as an explanatory paradigm for cause and effect pathway used for understanding biologic systems, e.g., one gene one disease.

Dogma that health care equals health. Health care is an industry, health is a biologic state.

A strong societal belief that health/ill-health is somehow, and irrevocably, endowed to us via genes and thus any *changes* in health, throughout our lives, lie outside of our potential influence.

## Materials

The time period from 1960s to the present has been selected because it incorporates unprecedented socio-economic and scientific developments, events within the span of only two generational cohorts.

Taking research findings from various, even seemingly unrelated fields of study, is encouraged by systems science in order to look for isomorphism, answers that some fields already have while others are still searching for them or are just formulating questions; it supports the premise that various systems theories resonate and can be found in numerous, seemingly unconnected fields.

In addition to scientific articles, general public domain publications were also selected, especially ones describing characteristics of the larger societal system. The collected information was grouped by similarities with systems science principles. For example, for entropy, reports of decline and diminishing functionalities were extracted; for chaos, publications highlighting exponential excess of economic bubbles or unmitigated cellular growth, were mined. For systems in health territory, descriptions of optimal adaptation and evolution were examined.

Due to the scope of the research topic and the diversity of material used, some extracts are included for targeted review.

### Change

Every event, no matter how remote or long ago, echoes across all other events (Mandelbrot, 2004).

Set size and order effects decisions (Hills et al., 2013).

Fear transforms us in physiological ways, making us less able to take in and learn new information (Jha, 2013).

Risk of overdiagnosis exists (Editorial, 2013).

Informed choice in cancer screening (Welch, 2013).

Of the 57 cancer screening trials examined, the most important harms of screening-overdiagnosis and false positive findings-were quantified in only 7 and 4%, respectively (Heleno et al., 2013).

Global temperatures highest in 4000 years (Marcott, 2013).

Uncertainty—the other side of prognosis (Smith et al., 2013a,b).

Scientific uncertainty does not mean we know nothing… we need to embrace uncertainty, especially when trying to understand more about complex systems (Aigrain et al., 2013).

A decade that began with the “reality” television craze exemplified by “American Idol” and “Survivor”—both blissfully devoid of any reality whatsoever—spiraled into a wholesale flight from truth… [resulting in] two true national catastrophes, a wasteful war and a near-ruinous financial collapse (Rich, 2009).

The twenty-first century has presented some stunning challenges to the United States: The popping of the Tech Bubble, the attack on the Trade Towers, wars in Afghanistan and Iraq, Hurricane Katrina, the collapse of residential real estate, the Financial Crisis, the Oil Catastrophe in the Gulf of Mexico, the outing of the 1%, the Fiscal Cliff debacle, etc. (Short, 2013).

We are into the… phase… where fear, lack of policy options, and loss of control can dominate relationships (Gross, 2011).

Data are unconnected “facts”; information represents data that have been fitted into categories and patterns; knowledge derives from information (Toffler, 1990).

### Systems

A cell has to have a size appropriate to its position within the overall tissue… cells can measure their own size and regulate the timing of cell division accordingly… possibly by reading out intracellular gradients… mechanical properties of the cell surface and of cytoskeletal elements (microtubules) (Marshall et al., 2012).

Cytoskeletal proteins, arbitrators of neuroplasticity, in particular microtubules [used for] information processing, are dysfunctional in mental illnesses… neuroplasticity is compromised (Woolf et al., 2010).

The key to a healthy life is organization… cells possess an innate ability to self-organize into communities… these communities of different types of cells can also organize themselves… to form and maintain healthy tissue. As new cells replace old ones… the architecture of that specific tissue must be maintained. Otherwise, cancer or other diseases can arise… Cells that properly organize themselves into communities live long and prosper, whereas disorganized cells can become cancerous (Chanson et al., 2011).

Contractility of boundary [of] a system is related to its semipermeability and the balance of extracellular and intracellular (forces) (Bauer and French-Constant, 2009).

### Networks

Visual surroundings are… crowded with information… The brain automatically detects and biases attention toward important and valuable features… two regions—the ventromedial prefrontal cortex (vmPFC) and the anterior cingulate cortex (ACC)—are involved in guiding attention to the most valuable objects in a scene… the ACC is connected with brain areas involved in directing eye gaze and planning other movements, and the vmPFC shares connections with areas that are critical for memory and emotions (Weaver, 2011).

Every time our bodies record an experience… the essence of who you are is stored as synaptic interactions in and between the various systems of your brain… activity induces growth (LeDoux, 2003).

What you see can override what you hear… vision is influencing the hearing to change your perception of reality… brain is intrinsically unreliable… one extra spike affect[s] millions of neurons… each neuron connects to about 10,000 others, resulting in over 8 million kilometers of wiring in the human brain (London et al., 2010).

The brain considers both sight and sound when processing speech. However, if the two are slightly different, visual cues dominate sound; neural signals in the brain that should be driven by sound are being overridden by visual cues (Smith et al., 2013a,b).

Humans and birds have brains that are wired in a similar way… for high-level cognition such as long-term memory and problem solving, a capacity for complex social reasoning, and some even use tools… hippocampus (important for navigation and long-term memory in both birds and mammals)… [has] very dense connections to other parts of the brain in both… the prefrontal cortex in mammals (important for complex thought such as decision making) [and] nidopallium caudolaterale has a similar role in birds (Gunturkun et al., 2013).

Alcohol reduced the coupling between the amygdala and the orbitofrontal cortex, an area of the prefrontal cortex implicated in socio-emotional information processing and decision-making… alcohol reduced the reaction in the amygdala to threat signals (Gorka et al., 2013).

Hearing loss [leads to] cognitive decline in older adults (Lin et al., 2013).

Smell [loss as an early sign of] degenerating brain (Doty, 2013).

After exercise [there are] epigenetic modifications… DNA within skeletal muscle bears fewer methyl groups (Barrès et al., 2012).

Physical exercise of the professional athletes [activates]… telomerase and stabilizes the telomere (Werner et al., 2009).

With an estimated 86 billion neurons and about a trillion synapses per cubic centimeter of cortex, the human brain is arguably the most complex system in the human body, and it is the seat of diseases and disorders that affect an estimated one billion people worldwide (Herculano-Houzel, 2009).

[There is] striking differences in the neural wiring of men and women… the “connectomes” of the sexes… greater neural connectivity from front to back and within one hemisphere in males, suggesting their brains are structured to facilitate connectivity between perception and coordinated action… in females, the wiring goes between the left and right hemispheres, suggesting that they facilitate communication between the analytical and intuition… the opposite prevailed in the cerebellum… [only] a few gender differences in the connectivity in children younger than 13 years, but the differences were more pronounced in adolescents aged 14–17 years and young adults older than 17… Females outperformed [on psychological tests] males on attention, word and face memory, and social cognition tests. Males performed better on spatial processing and sensorimotor speed. Those differences were most pronounced in the 12–14 age range (Ingalhalikar et al., 2013).

[Synapses have] a preferred/optimal frequency for maximal learning [that] needs to be rhythmic [but] learning/synaptic activation pattern is temporary-at a given frequency/rhythm. There is an optimal brain rhythm/frequency, for changing synaptic strength; each synapse is tuned to a different optimal frequency for learning (Kumar and Mehta, 2011).

The capacity of synapses to preserve their specific properties might be more limited than previously thought, raising questions about the long-term reliability of individual synapses (Minerbi et al., 2009).

Vertebrate synapses have about 1000 different proteins, assembled into 13 molecular machines, one of which is built from 183 different proteins… each region uses different combinations of the 1000 proteins to fashion its own custom-made synapses… The human brain has about 100 billion neurons, interconnected at 100 trillion synapses (Emes et al., 2008).

Between 3 and 300 milliseconds is the range of time [that] is involved in many aspects of cognition… [For example] the response time while driving a car is around 300 milliseconds (Nolte, 2001).

Median latency of 22.8 years [for mesothelioma to develop following asbestos exposure] (Frost, 2013).

DNA methylation age… [of] 20 cancer types exhibit[s] significant age acceleration, with an average of 36 years. Low age-acceleration… is associated with a high number of somatic mutations and *TP53* mutations, while mutations in steroid receptors greatly accelerate DNA methylation age in breast cancer (Horvath, 2013; Verhoeven et al., 2013).

DNA methylation… [becomes] highly dynamic in brain cells during the transition from birth to adulthood… [there is] widespread reconfiguration in the frontal cortex of mouse and human [with] synapses… growing rapidly… About 80–90% of CpG sites (cytosine, guanine), are methylated in human DNA. … DNA methylation can also occur [as] “non-CG methylation” (cytosine, guanine)… [which] accumulates in neurons through early childhood and adolescence, and becomes the dominant form of DNA methylation in mature human neurons (Lister et al., 2013).

DNA methylation age measures the cumulative effect of an epigenetic maintenance system, epigenetic clock… [and is] close to zero for embryonic and induced pluripotent stem cells… it correlates with cell passage number (Horvath, 2013).

Epigenetic mechanisms are critical for… brain patterning, neural stem cell maintenance, neurogenesis and gliogenesis, neural subtype specification, and synaptic and neural network connectivity and plasticity (Qureshi and Mehler, 2011).

Gene mutations caused by a father's lifestyle can be inherited by his children, even if those mutations occurred before conception (Linschooten et al., 2013).

Osteocalcin… secreted by osteoblasts… [is] involved in… bone-to-brain signaling [it]… binds to neurons in the brainstem, midbrain, and hippocampus [and] promotes the birth of neurons… [it also] increases the synthesis of several neurotransmitters (serotonin, dopamine, and catecholamine)… osteocalcin must act during development… [it] crosses the placenta from mother to fetus… this maternal pool of osteocalcin is necessary for formation of the hippocampus and the establishment of memory… children born from undernourished mothers [who] have low bone mass, which affects osteocalcin production, [often develop] metabolic and psychiatric disorders (Oury et al., 2013).

Good Bacteria Arrive from Mum's Gut Via Breast Milk… bacteria can travel from the mother's gut to her breast milk… same strains of *Bifidobacterium breve* and several types of *Clostridium* bacteria… Strains found in breast milk may be involved in establishing a critical nutritional balance in the baby's gut (Jost et al., 2013).

Telomere length measured toward the end of the growth period (in avian species) [is]… the strongest predictor of lifespan… short telomeres at any age are associated with an increased risk of death (Monaghan, 2012).

Low literacy in pre-teen girls strongly predicts childbearing among US teens… girls with a less-than-average reading skill were 2.5 times more likely to have a child in their teen years (American Public Health Association, 2012).

Memory [represents] a reconstruction of… experiences on the basis of the way they were stored, not as they actually occurred… the brain that does the remembering is not the brain that formed the initial memory… remembered experience is a distortion of actual experience (LeDoux, 2003).

Memories can be unreliable (Ramirez et al., 2013).

Nutrients and their metabolites influence the epigenome… [through] epigenetic-modifying enzymes… most cancer cells exploit metabolic pathways for their hyperproliferative activity (Hino et al., 2013).

We are in reality diverse beings in that a single person is genetically not a single entity… Having multiple genotypes from mutations within one's own body is somewhat analogous to chimerism… Most genetic changes don't cause disease (Samuels et al., 2013).

Amygdala… controls defensive responses… amygdala also can be activated directly from the thalamus… bypasses the neocortex, it only provides the amygdala with a crude representation of the external stimulus… cells in the lateral amygdale respond to the information directly from the thalamus faster that they can respond to info from the cortex… (LeDoux, 2003).

The dorsal thalamus is a sensory gateway of the brain that receives visual, somatosensory, and auditory information. Thalamocortical axons convey this sensory information from the dorsal thalamus to the cerebral cortex and hence are essential to brain function (Lokmane and Garel, 2011).

The sympathetic nervous system… “talks” to cells in various organs throughout the body. When the sympathetic nervous system is activated… during stress, it communicates with receptors on cells through the release of neurotransmitters… norepinephrine and neuropeptide Y (NPY)… breast cancer cells express the receptors for NPY… [which] accelerates cell growth as well as cell migration (Kimmerl, 2010).

Epigenetic mechanisms are critical for orchestrating nearly every aspect of neural development and homeostasis… brain patterning, neural stem cell maintenance, neurogenesis and gliogenesis, neural subtype specification, and synaptic and neural network connectivity and plasticity (Qureshi and Mehler, 2011).

### Relationships

Kinesins are the railway engines of the cell, hauling molecular cargo over long distances along microtubule tracks. The kinesin-microtubule railway system is central to the self-organization of eukaryotic life (Cross, 2010).

Multicellular organisms have certain advantages over those that are single-celled. To evolve, however, they must… ensur[e] that their constituent cells cooperate with one another… A number of genes were identified of which knockdown allowed competitive behavior to dominate. These genes formed a network centered on p53, topoisomerase 1, and olfactory receptors (Dejosez et al., 2013).

Relationships must involve ethics/morality (generally accepted rules/social contract)… When a relationship reaches mistrust… old system must be dissolved and a new one built through “higher logic” than one fostering conflict (van Gigch, 2007).

A polarized political system seems unable to solve problems that involve trust (New York Times, 2010).

Brain is conducting an internal simulation as a way to understand the metaphor (Lacey et al., 2012).

Even before they are born, babies accumulate changes in their DNA through… DNA methylation that may interfere with gene expression, and… their health as they grow up… DNA methylation changes occurring early in life may have lasting impacts… Maternal BMI (prior to becoming pregnant; [there is] high proportion of obesity among women of reproductive age) (Herbstman et al., 2013).

### Flow

During sleep… genes [are] involved in synthesis of vesicles [for new] neurotransmitter[s]… (Pack, 2009).

Circadian clock… [also] controls the numbers of inflammatory cells… interleukin-17-producing CD4+ T helper cells (T_*H*_17)… if their numbers are not controlled properly… [it] can lead to [autoimmune] inflammatory diseases… [disruption of] normal day-night light cycles of mice… [leads to] too many T_*H*_17 cells and [they accumulate] in the intestines. As a result, these mice were more prone to develop an IBD-like disease [inflammatory bowel disease] (Yu et al., 2013).

The misalignment of an individual's internal [circadian] clock with its environment is associated with adverse health consequences, including metabolic disorders and cancers… feedback loops (cytosolic loops) are considered the prime mechanism sustaining intracellular rhythms (Rey and Reddy, 2013).

Sleep has a critical function in ensuring metabolic homeostasis… natural sleep or anesthesia are associated with a 60% increase in the interstitial space, resulting in a striking increase in convective exchange of cerebrospinal fluid with interstitial fluid… convective fluxes of interstitial fluid increased the rate of β-amyloid clearance during sleep… the restorative function of sleep may be a consequence of the enhanced removal of potentially neurotoxic waste products that accumulate in the awake central nervous system (Xie et al., 2013).

Circadian clock… [is located] in the suprachiasmatic nucleus (SCN) of the hypothalamus… and liver, fat, heart, and lung… [it is the] primary light sensing mechanism… in the retina… [it] involves the pigment melanopsin in retinal ganglion cells… This master clock in the SCN communicates with the peripheral clocks… 2000 genes [are] either turned on or off during sleep—a major purpose of sleep is to rebuild the molecules that are essential for cell function… the speed of recovery is an indication of system robustness… all aspects of the unfolded protein response occur after 6 h of sleep deprivation in the mouse brain… [and] leads to reduced protein translation… cellular stress may be a factor in neurodegenerative disorders… The shift worker… shifted eating schedules, and [has] sleep deprivation… sleep/wake cycle and clock mechanisms are desynchronized… [consequential] medical problems… [include] an increased risk for heart disease and some forms of cancer (breast and prostate) (Pack, 2009).

Sleep helps… memory consolidations regarding motor memory learning (Tamaki et al., 2013).

### Complexity

“Pluralistic ignorance”… [implies that] a large proportion of a population misunderstands reality. They may all agree, but they are, nonetheless, mistaken (Wade, 2010).

A collective mind is a terrible thing to lose… Congress cracks up (Collins, 2013).

Senate is “broken,” said Harry Reid, [Majority Leader] (Weisman and Peters, 2013).

Mixing ignorance and democracy (Chapman, 2012).

One in 3 Americans failed to return census forms (Roberts, 2010).

The single biggest impediment to a stronger economic recovery has been the years of dysfunction in Washington and the policies that have emerged (Packer, 2013; Rattner, 2013).

### Output/emergence

Believe in evidence… Evidence is evidence (Gitschier, 2013).

Success/Expert [emerges from] 10 years/10,000 hours of purposeful training/internal motivation… [is strongly related to] the quality and quantity of practice… Experts [have the ability] to free up attentional resources… Attention is a resource with severe capacity limitations (Syed, 2010).

There are no instant experts in chess… a master has spent perhaps 10,000 to 50,000 hours staring at chess positions (Chase and Simon, 1973).

Behavioral economics [explore] how people misinterpret information, how their emotions distort their decision, and how they miscalculate probabilities (Mandelbrot, 2004).

The paradigm that we use filters/affects what we perceive/see and hear (Berger and Ehrsson, 2013).

Facts from 360 B.C.–A.D. 2012… have finally died (Huppke, 2012).

Cognitive ability is related to… behaviors that affect health… adolescents scoring high on the cognitive ability test have healthier dietary habits and engage more often in physical activity (Junger and van Kampen, 2010).

Vigorous physical activity… can protect individuals from the effects of stress by reducing its impact on telomere length (Puterman et al., 2010).

Stress makes its molecular mark on epigenetics (Nester, 2012).

Adversity is toxic to telomeres (Blackburn and Epel, 2012).

People with recurrent depressions or those exposed to chronic stress exhibit shorter telomeres in white blood cells… oxidative stress and inflammation accelerate this shortening. Telomere length… has been linked to age-related diseases, unhealthy lifestyle, and longevity. Shorter telomere length is associated with both recurrent depression and cortisol levels indicative of exposure to chronic stress (Wikgren et al., 2011; Cohen et al., 2012).

In 1985 most people said they had three close friends. In 2004 the most common number was zero (Lieberman, 2013).

GABA neurons are particularly susceptible to oxidative stress (Yowtak et al., 2013).

An unhealthy lifestyle leaves traces in the DNA… [via] methylation (Petersen et al., 2013).

Telomeres… reflect the history of oxidative stress… smoking, unhealthy foods, extreme physical or mental stress shorten telomeres… shortened telomere shows what you have done to/with Life (Barrett et al., 2012).

Cognitive ability is related to health and mortality (Junger and van Kampen, 2010).

Research on animal thinking—“cognitive ethology”… bat echolocation… other species are likely to have mental lives very different from ours. They see the world very differently and probably think very differently about it as a consequence (Rendall, 2013).

Human cognition shapes foreign and defense policies… cognitive and methodological challenges faced by analysts can lead to intelligence failure… what mattered wasn't just the evidence… [but] the views, biases and organizational flaws of the analysts could often have a huge bearing on their interpretations… “prevailing beliefs” can act as a “filter” for both supporting and contradicting information; how the principle of “availability” leads even well-trained analysts to interpret information in light of what is on their minds at the time, and how analysts can be guilty of “layering”: uncritically piling new evidence on top of old. These types of “cognitive biases,” in addition to problems posed by sources and the intense pressure analysts are under, can all contribute to intelligence failures (Wirtz, 2013).

US housing bubble was estimated to be ×1/10,000 year event (Grantham, 2007).

### Dynamic systems model

#### Chaos

Lifestyle changes affect telomerase activity and telomere length (Ornish et al., 2013).

Patients with serious mental illness are 2.6 times more likely to develop cancer than the general population (McGinty et al., 2012).

Increased metastasis to the lung have been observed after acute bacterial infection (Smith et al., 2013a,b).

Expressions of immunoregulatory genes… [are] reduced in patients in the early phase of sepsis… non-survivors showing a significantly greater reduction than survivors (Parnell et al., 2013).

[Markers of systemic inflammation can assume] independent prognostic value in patients with a variety of cancers (McMillan, 2013).

Women's breast tissue accrues methylation [as part of epigenetic clock]… breast cancer tissue appeared to be an average of 12 years older than other tissues in the body… [and] tissue from 20 [other] cancer types looked an average of 36 years older than healthy tissue… methyl groups can selectively switch-off genes (Horvath, 2013).

[Autonomic nerve fiber system] regulates prostate cancer development and dissemination in mouse models… human prostate adenocarcinoma specimens… revealed that the densities of sympathetic and parasympathetic nerve fibers in tumor and surrounding normal tissue were associated with poor clinical outcomes (Magnon et al., 2013).

[There is a] close association among reactive oxygen species, chronic inflammation, and cancer (Gupta et al., 2012).

Cancer—due to enhanced resistance to cell death and neurodegeneration—due to premature cell death… disease mechanisms at opposite ends of a spectrum… Accumulating evidence… link these two disparate processes… neurodegenerative disorder[s] have a reduced incidence for most cancers… (Alzheimer/AD)—60% reduced risk of cancer, and a history of cancer—30% reduced risk of AD… but an increased risk for… (malignant melanoma)—[Parkinson's /PD] (Plun-Favreau et al., 2010).

#### Entropy

Misfolded proteins can cause various neurodegenerative diseases (Tetrakis et al., 2012).

Aging impairs the unfolded protein response to sleep deprivation and leads to pro-apoptotic signaling (Naidoo, 2008).

[Dietary vitamin A, through its metabolite retinoic acid] converts glutamate to the inhibitory neurotransmitter GABA… [in a deficiency, it] greatly diminished GABA… Deficiencies in GABAergic neurons [are]… associated with… Huntington's disease, autism, schizophrenia, and epilepsy (Bravo et al., 2011; Chatzi et al., 2011).

Bilingual patients developed dementia 4.5 years later than the monolingual ones… also in illiterate patients (suggesting that education is not a sufficient explanation for the observed difference) (Alladi et al., 2013).

How institutions decay and economies die through degeneration (Ferguson, 2013).

In Alzheimer's disease, [there is] accumulation of beta amyloid within synapses (Funk et al., 2011).

Age-related dementia is likely the result of a declining ability of neurons to dispose of unwanted aggregated proteins (Schipanski et al., 2013).

Modifiable risk factors for Alzheimer's disease are… physical inactivity, depression, smoking, mid-life hypertension, mid-life obesity, low education, and diabetes (Barnes and Yaffe, 2011).

Brain-derived neurotrophic factor (BDNF)… impact[s] neuronal survival and function and improve[s] synaptic plasticity and long-term memory. Circulating BDNF levels increase with physical activity and caloric restriction… lower circulating BDNF [have been observed] in persons with Alzheimer disease (Weinstein et al., 2013).

Handwriting as an objective tool for Parkinson's disease diagnosis (Rosenblum et al., 2013).

Nearly 18% of those with PD [Parkinson's disease] were deficient in vitamin D [which correlate[d] with] severity of disease (Ding et al., 2013).

Risk of cancer was cut in half for people with Alzheimer's disease and the risk of Alzheimer's disease was reduced by 35% for people with cancer (Musicco et al., 2013).

Neurodegenerative and psychiatric disorders are considered to be synaptopathies… synaptic vesicles… store neurotransmitters within… [but] synaptic vesicles must be… refilled (Armbruster et al., 2011).

Depression may be an independent risk factor for Parkinson's disease… People with depression were 3.24 times more likely to develop Parkinson's disease than those without depression (Shen et al., 2013).

Nerve cell body death represents the final event of [neurodegeneration]… protecting cell bodies from death has no impact on disease progression whereas blocking preceding axon breakdown has a significant benefit… During early development, axons are pruned to ensure normal growth of the nervous system. … this pruning process becomes reactivated in neurodegenerative disease, leading to the aberrant loss of axons and dendrites. Axonal pruning in development is significantly influenced by (caspase-3 and caspase-9)… [which] induce axonal degeneration… their action is suppressed by a protein XIAP (X-linked inhibitor of apoptosis)… [the balance] between caspases and XIAP… may shift during neurodegenerative disease (Unsain et al., 2013).

Oxidative stress reflects an imbalance between the systemic manifestation of reactive oxygen species [ROS] and a biological system's ability to readily detoxify the reactive intermediates or to repair the resulting damage. In humans, oxidative stress is thought to be involved in the development of cancer, Parkinson's disease, Alzheimer's disease, atherosclerosis, heart failure, myocardial infarction, fragile X syndrome, Sickle Cell Disease, lichen planus, vitiligo, autism, and chronic fatigue syndrome. The major portion of long-term effects is inflicted by damage on DNA (Evans and Cooke, 2004).

Our brain has not evolved to the point where the new systems that make complex thinking possible can easily control the old systems that give rise to our base needs and motives, and emotional reactions… doing the right thing doesn't always flow naturally from knowing what the right thing to do is… the self is maintained by systems that function both explicitly and implicitly (LeDoux, 2003).

Obesity is an inflammatory disease (Lim et al., 2013).

## Methods

Three systems-related methodologies were used in this study: Systems Science, Dynamic Systems Model, and the Kondratieff's Long Wave cycle. Each approach offers a unique but complementary perspective on examining *change* and its risk/uncertainty relationship that impacts all involved systems; all three methodologies offer a framework for visualizing and understanding life of biologic entities, its harmony or disharmony, as well as gauge the risk and uncertainty of *change*.

Systems science methodology is pertinent to this study because it describes the characteristics of living systems: Systems have components/sub-systems, from cells to societies, which should be numerous and variable but with a high degree of shared decision rationality (based on current general knowledge of physics, biology, ecology, etc.). Systems have relationships with feedback loops which, in healthy systems, express reciprocity, fairness, cognition-dependent empathy, and trust. Relationships create functional complexity which produces eventual outcome, system's emergence. When some of the above-listed features are absent, the gaps serve as a warning of potential instability and fragility of such a system.

The term, complex adaptive system, summarizes the positive attributes of a healthy system that is capable of producing value, its emergence, through organized complexity. Any disharmony in relationships has the capacity to *change* organized into disorganized complexity and the likely consequential absence of value creation, a portrait of an unhealthy system. Complexity has a major impact on the system's capacity to manage *change*. The significance of maintaining a state of health of any system is *prima facii*. Healthy human body is the best known complex adaptive system composed of numerous smaller sub-systems, all the way to cells, microorganisms, viruses, etc. Complex adaptive systems cannot be micromanaged and successfully live; they have to be optimized through complementary self-organization of components and governing hierarchy in order to achieve organized complexity.

Gradient flow of energy and information, within a function-defined size, shape, and boundary, is essential to the survival of any biologic system. It refers to the intake/throughput/output sequence that creates a directional and proportionate balance from intake to output; energy as well as information intake have to be managed to maintain such a flow; obesity may be used as an example where intake greatly exceeds output resulting in abnormal throughput/metabolism and accumulation of unprocessed energy; similarly, unfiltered intake of information overwhelms the throughput making rational output/decisions difficult; a common communication platform enables inter-operability. Optimized systems, those in health territory, exhibit flow with gradient balance; it has forward/output bias, allowing for both multiplication and differentiation of system's components. In the zone of chaos, the flow becomes exponential and output-focused where energy is being used mostly for multiplication but without differentiation. In the zone of entropy, the flow is diminished with near zero gradient; no multiplication or differentiation is observed.

Utilizing systems science for evaluation of *change* transforms the traditional methodology of establishing linear probability of outcome into a multidimensional/non-linear/fractal contextuality. Such an approach offers different and likely more robust interpretation of what is happening and how best to respond.

System's components should be numerous, variable, and evolvable; boundary needs to be semipermeable; systems' size should reflect balance between function and structure, one that allows for oscillation with cycles. Systems should demonstrate system-within-a-system patterns of self-affinity and self-similarity of smaller and larger systems; fractal patterns that such systems generate can be considered a reflection of adaptation and evolution.

Complexity, arising from optimizing relationships, incorporates processes of self-organization within horizontal hierarchy (“people in the trenches”) and governing vertical hierarchy (creates laws, their enforcement, institutions, tariffs, etc.). Organized/optimizing complexity gives rise to collective intelligence encompassing collective rationality and responsibility; a potential for creating value/its emergence, is present; such a system is robust enough to express high degree of resiliency and functional redundancy. Lack of organized complexity, expressed as disorganized complexity, leads to absence of value creation and cognitive dissonance/stress.

When Kondratieff described the cycle that bears his name in the 1920s (Kondratieff, 2010), he followed only the fluctuations of commodity prices and credit. This Long Wave is a graphic expression of *change* in the larger socio-economic system, which in this research, has been modified to reflect fluctuations of societal trust mirrored in credit-worthiness. The average time span, 50 years, also includes two generational cohorts (Strauss and Neill, 1991), each with its own culture dominated by differing attractors.

The connection, between the Long Wave credit cycle and changing societal trust, is visualized as follows: economy equals societal relationships which are always based on variable level of trust reflected in the fluctuating level of worthy credit. When trust diminishes so will solid credit. Also, the word credit is derived from Latin word *credo* which means belief/trust.

Dynamic Systems Model (Janecka, 2007) complements Systems Science because it places a given *change*-generating system and any contextually-related systems, in a multi-dimensional evolving pattern. Such a mosaic allows for a more accurate creation of risk/uncertainty ration because both risk and uncertainty vary with system's position within the Model and the Long Wave Cycle.

The Model has defined zones based on their functionality: The Health Territory indicates optimal functioning of a system. It dynamically spans the boundaries of two neighboring zones, the outer core of Entropy and the inner edge of Chaos. Extremes, the outliers in this Model, include the outer edge of Chaos and the inner core of Entropy. Each classification within this Model reflects, on one hand, the degree of system's capacity for organized complexity, adaptation, and evolvability as well as the ability to produce positive emergence/value; on the other hand, the Model also reveals the high likelihood of random events or system entropic end-phase. Health Territory produces evolutionary changes; Chaos generates revolutionary *changes*.

When a system is in Health Territory, random events are rare; most randomness is absorbed/dealt with proactively by a system that is fit; because of infrequency of randomness, it is possible to anticipate it only as “possible”/unlikely event.

When a system is in Chaos, randomness is, however, much more frequent/the norm, the time frame is short, incidence is frequent (e.g., tech bubble followed by real estate bubble followed by financial bubble-all within 7 years: 2000–2007). Events in Chaos may lead to anarchy (summation of randomness and asynchronous cycles); acceleration of DNA methylation can be observed and measured demonstrating rapid cellular aging.

## Results

The following research questions were explored:

What is *change* from systems science perspective?

How can *change* be differentiated into risk and uncertainty?

Can systems science provide clues as to why identical *change* may have variable impact?

Is there a broad measure of societal trust that impacts *change*?

*Change* is always multidimensional and, except for laboratory experimentation, is never fully determinate. *Change* comes from altered network relationships and, in turn, alters them back. Systems science perspective improves the odds of understanding *change.*

*Change,* from systems science perspective, is an output/an emergence of a given system; it represents the culmination of inter- and intra-system's relationships that create the character of its complexity. Systems science offers a framework to ascertain the degree of synch among inter-related biologic systems. Relationships determine the character of system's complexity and its capacity for creation of an optimizing output as well as the competence to successfully absorb even non-optimizing inputs. Study observation: A minority of societal systems are harmoniously related to systems science principles.

C*hange* can be differentiated into risk and uncertainty; risk is quantifiable by our primary or expanded senses; the rest is uncertainty. Study observation: The reliance on senses for primary filtering of *change*-derived input has been greatly diminished in the societal system; it has been delegated to technology but without parallel enhancement of cognition-dependent knowledge creation.

Identical *change* may have variable impact depending upon the degree of compliance with systems science principles of both the originating and *change*-receiving systems. A *change*-assessor is also viewed as a system with a specific hermeneutic paradigm.

For each *change*, a systems science-based analysis should focus on the system that generated the *change* as well as the ones that are impacted by it. Three features are key: 1-the character of their complexity, 2-the type of relationships, and 3-the emergence. Such observations allow topological placement of any system within the Dynamic Systems Model, either in the optimal Health Territory or non-optimal zones of either Chaos or Entropy.

Diseases reveal cascade of *changes* taking place within a bodily system. They mirror altered expressions of morphologic phenotype driven mostly by *changes* in the epigenome which was misregulated, often by decisions. Such decisions follow imbalance of energy and information flow through the synaptic neuro-net affecting its directionality as well as the variability of functional states of either excitation or inhibitions. Biologic systems maintain synaptic flow via sensory input. When the richness of input begins to fade or throughput/metabolism is impaired, network starts to regress and the system enters entropy.

Stress desynchronizes neuro-net from its dependence on cycles, creating dissonance. Study observation: Most corrective measures that are being utilized to resolve the dissonance, by individuals and collectively by society, have had mostly downstream/symptoms focus.

The characteristics of a system's existential state are identifiable by exploring the following statements: (a) complexity is system's functionality; it can be observed as organized/optimized complexity or a disorganized/non-optimized; each functional path determines the eventual outcome/output/emergence, either as value or its absence; (b) relationships determine system's complexity; optimizing relationships are reciprocal, fair, empathic, and are based on trust; (c) cognition reflects the state of system's synaptic neuro-net and generates decisions; conscientious effort carries out optimizing decisions. All systems are under the influence of cycles, internal and external ones; working against cycles is to systems' detriment as it generates stress.

Study observation: Most studied systems were found to exist with a profound lack of reciprocity/fairness and empathy in their relationships on societal and global levels with paucity of optimized decisions; generated outcomes have been observed to emerge from the prevalence of disorganized complexity, non-optimizing outputs, and poor resiliency toward *change*; trust has been grossly absent. Highlights: Obesity and inactivity are predominant on all societal levels, memories are failing an increasing percentage of the population, and wars continue as expressions of failing relationships. Credit has changed into “debt based on debt” on a massive scale accompanied by morphing of trust into distrust. Many decisions even threaten societal survival. Organized complexity seldom exists and, as a consequence, value has rarely been created during the studied period.

Trust is the key to sharing risk; no societal system or a medical team can optimally function without it. Trust creates a foundation for optimized relationships and exchanges that can lead to the creation of organized complexity with hallmarks of adaptation, evolution, and value creation.

Study observation: Vanishing trust and mushrooming uncertainty in a society exhaust the limited reservoir of cognitive capacity that exists to make rational, risk-based decisions, and leads to either poor or no decisions at all. As a consequence, there is a diminishing ability to lead, achieve consensus, make facts-based decisions; logic vanishes, and emotions surge. With absence of common sense, societal *changes* become mostly reflection of uncertainties; social bonds fragment in spite of knowing that freedom is strongly connected to trust.

Study observation: Societal trust is difficult to measure. A proxy can be adopted from the financial markets which document, on minute to minute and long-term bases, the state of flow of credit on a very large scale because the amount and quality of credit is tied to trust; the time periods, alternating between when credit is and is not based on trust, show significant fluctuations that can be charted by the Kondratieff Long Wave. The Long Wave is a graphic expression of *change* in the larger socio-economic system, oscillating from risk-based trust to uncertainty-based credit. Without trust, what was originally categorized as risk becomes uncertainty.

Lack of trust forces people to regress from Maslow's “sense of belonging” level of human needs back to the basic, ground level, of “safety and security” (Maslow, 1943, 1954).

Clusters form in response to attractors that claim dominance over awareness generated by synaptic network. Study observation: Diseases preferentially cluster in various zones of the Dynamic Systems Model, often in opposite zones of Health Territory: cancer in chaos and degeneration/chronic inflammation in entropy; the first is expected to have excess of synaptic excitation and the second dominance of inhibition. One disease may potentiate or at least be associated with the occurrence of another that is often found in the same zone, e.g., mental illness is often accompanied by increased incidence of cancer. However, other diseases, which belong to differing zones (Chaos vs. Entropy), appear to lessen the development of those in contrary zones: neuro-degeneration in Alzheimer's or Parkinson's diseases show significantly lower association with cancer incidence. Topologic placement of various diseases into the Dynamic Systems Model can be utilized for further learning (diagnosis, treatments, etc.) especially in cases where advanced knowledge of some diseases is already available and can be judiciously explored in diseases still needing solutions.

Study observations point toward the dependence of a living epigenome on its ancestral generations and the time window during which it can be sufficiently altered by choices: Gestation and birth reflect the morphologic steps taken by a new bodily system to achieve a certain phenotype following instructions received from ancestral epigenomes and the influence of maternal bodily system during pregnancy. Three Life Phases can be charted: The first phase of life, about 25+ years, is named an Ancestral Phase in this study in order to reflect the implementation of accumulated epigenetic *changes* from previous generations. The second phase is labeled a Phase of Decisions where the now-adult may exert intentional modifications on its evolving epigenome through decisions and choices; the third phase, from age 50+ years on, is the Phase of Consequences, with primary influence taking place by a pre-set epigenome formatted during the second life phase. A key risk exists during the teen years of the first, ancestral, phase, because if this evolving youngster conceives a yet another generation prior to its ability to correct any epigenetic malfunctions received from the forebears, the misregulated epigenome will continue.

Study observation: Extraordinary accomplishments have been achieved by some societal sub-systems in the fields of genomics, planetary exploration, and quantum physics indicating functioning optimized smaller systems that can exist within a larger non-optimized system.

## Discussion

### The concept

*Change* is generated by a system and affects other systems; thus, knowledge of systems, offered by systems science, is paramount. Not all systems are alike; what differentiates them are relationships arising from networks which must be sustained by a gradient flow of energy and information; Dynamic Systems Model allows for visualizing such differentiations (Figures 1A–F). Not all *change* is discernible but a great degree is via senses and is considered risk; uncertainty exists outside of sensory perception. All systems are engaged in inter-relationships with other systems and exert variable mutual influence; larger systems wield stronger influence. The Long Wave, charting expansions and contractions of credit markets over decades, also reflects reciprocal fluctuation of trust that exists within the large socio-economic system; and, trust is the key to forming systems relationships that characterize all systems.

**Figure 1:** **(A)** Zones of dynamic systems model. **(B)** Composition of Health Territory. **(C)** Characteristics found in Health Territory. **(D)** Characteristics found in Chaos. **(E)** Characteristics found in Entropy. **(F)** End-state features of Chaos and Entropy as well as feasible corrective steps.

### Expanded concept

Understanding c*hange* needs context; without it, randomness prevails as no system can exist in isolation. The context for understanding includes: Function and structure of biologic systems within their networks as each generates its own output/emergence. Relationships exist as forms of flow of energy and information among networks creating complexity. The overall biologic system's output/emergence is a composite of yields of all the sub-systems and becomes new *change*, exerting influence, both, in reverse, on all of its sub-systems' networks via feedback loops, and, propagating forward, affecting all inter-related systems (Figures 2A–E).

**Figure 2:** **(A)** Schema of propagating *change* through functional and structural levels of a biologic system. **(B)** Propagating *change* paths. **(C)** Options that may activate system's paths. **(D)** Alternatives that may be present at system's paths. **(E)** Initiation of system's processes and selection of options by cognition.

Biologic systems are open systems—with intake/throughput/output—engaging numerous and variable components in network relationships. A system's core lies with the functional integrity of its networks. *Change* is a system's emergence/output, either positive or negative, arising at multiple crossroads of network relationships.

*Change* simultaneously consists of risk and uncertainty, in variable but roughly definable (R/U) ratios. Within this construct, taking a quantifiable risk implies that the probability favors the anticipated outcome but leaving a “door” open to the possibility of some unanticipated and uncertain result. Risk goes hand in hand with probability and pragmatic confidence generating a degree of rational optimism; uncertainty is more aligned with nebulous possibilities and evokes fear. As risk and uncertainty are inseparable, systems science would not favor that they are studied in isolation regardless of the applied mathematical algorithm or the employed computing processing speed. *Change* reflects ebb and flow of multidimensional temporal relationships of probable risk and possible uncertainty, a range of probabilities within almost unlimited possibilities. Trust is the binding key for any subsequent sharing of *change* assessment. In medicine, not structuring the risk/uncertainty ration may lead to over-, under-, or mis-diagnosis in larger proportion than when the ration is constructed (Editorial, 2013).

Uncertainty is open-ended and without boundaries due to the absence of sensory-derived parameters. Fear is tied to uncertainty as it creates a cognitive overload; the often incalculable and disproportionate weight, given to all the possibilities, generates non-optimizing stress/cognitive dissonance; acting only on uncertainty is a speculation.

How *change* is received by a system varies depending upon the following scenarios: an optimizing incoming *change* promotes other systems' optimization and vice versa; a non-optimizing *change* is expected to be absorbed by an optimized system. Biologic systems' functional and structural characteristics allow for topologic placement of each within the Dynamic Systems Model which facilitates differentiation between a healthy/optimizing system and one that is not.

*Change* may trigger sensory activation, within a range of its sensitivity and specificity, which can separate a portion of *change,* labeled as risk, leaving the remainder as an uncertainty; a risk/uncertainty ration (R/U) is created. Senses with cognition, which is variable and conditional, determine the fluctuating proportions in the R/U and its interpretation.

An evolving *change* is neutral and without meaning, until it is assessed in reference to some scale; considering the inescapable influence of the observer on the observed, conceptualized by Heisenberg (1949) and very broadly considered an extrapolation in this context; in this text it refers to the fact that our observations discard most of what *change* encompasses and what could be observed. For a signal to become data that leads to information, it must be first selected by a “collector,” be it a human or a programmed instrument; even at the point of “collection,” data and information are not neutral and are all subject to a form of uncertainty principle and the role of the observer. It is the selection and the connection of the dots/data which creates information and carries a strong subjective bias; what it means ends in the province of knowledge created by cognition; healthy systems benefit from optimizing *change* and modify most non-optimizing ones; vice versa scenario exists as well.

Similarly to Heisenberg's uncertainty principle, engaging at a systems' input, mentioned above, at the end point of attempting total understanding of *change,* it runs against Gödel's Incompleteness Theorem: “*all logical systems of any complexity are, by definition, incomplete*” (Casti and DePauli, 2001). Gödel's indeterministic principle is harmonious with systems science, broadly interpreted in this study as meaning that you can never measure and control all of system's variables; measuring some variables should acknowledge that knowing “some” is not necessarily representative of the whole.

*Change* reflects system's level of fitness; a healthy system is resilient, a pre-requisite for adaptation and evolution. Fitness significantly contributes to the maintenance of physiologic levels of cellular apoptosis/autophagy/necrosis and the level of telomerase, as well as their metaphoric counterparts in larger healthy systems. It would be highly unlikely for an unfit system to be capable of creating organized complexity that leads to value. Fitness is recoverable as Ornish demonstrated with groups of unfit patients through lifestyle *changes* (Ornish et al., 2013).

A flow of energy and information sustains systems' networks that generate and respond to *change*. The energy component is a product of a metabolic network; digested food manipulates gut microbiome which in turn influences neurotransmitters within a synaptic network (Ahn et al., 2013; Cotillard et al., 2013). Exercise develops and maintains the density of neuro-muscular junctions, the connectome, which shows various ratios of muscle fibers per nerve-endings; in early stages, neuro-degeneration impacts neuromuscular junctions, especially of the fine and fast muscles with the greatest density (intrinsic muscles of the hand, vocalis, and orbicularis occuli muscles).

Biologic systems, with their infinite and always transforming variables, are difficult to study; many specific tools are yet to be developed. Mathematical expressions of risk, uncertainty, optimism, fear, trust, etc. are seldom all encompassing. A comment, attributed to Albert Einstein, reflects the gap: *“As far as the laws of mathematics refer to reality, they are not certain; and as far as they are certain, they do not refer to reality”* Albert Einstein (Isaacson, 2008).

Similarly, several decades ago, another Nobel Prize winner, Frederic Hayek, warned that [there are] “*inherent limitations of our numerical knowledge*” (Hayek, 1974).

More recently, Heinz Pagels, a particle physicist at Rockefeller University, opined: “quants” [that] do quantitative finance [are] seduced by a vision of mathematical elegance underlying some of the messiest of human activities [and] apply skills they once hoped to use to untangle string theory or the nervous system to making money (Pagels, 1989).

Basic biologic systems (e.g., cells) can serve as examples of inter-dependability between function and structure that permeate all healthy systems; a structure, existing within a certain range and with a foldable framework, allows for flexibility/plasticity with a boundary that is semipermeable (Woolf et al., 2010; Chanson et al., 2011; Marshall et al., 2012).

The character of *change* is the reflection of system's topologic location within the Dynamic Systems Model which allows for categorization of systems to healthy and unhealthy ones, from societal to individual bodily systems. For example, a large societal system that functions within the Health Territory, demonstrates great capacity for collective intelligence with features of collective rationality and collective responsibility. Once such a system migrates into Zone of Chaos or Entropy, however, the collective intelligence rapidly diminishes. When such a system moves further and further into the periphery of Chaos, it reaches its “butterfly”/extreme stage which exhibits full breakdown of system's relationships with severe disconnect between horizontal and vertical hierarchy. Also, the frequency and severity of random events continue to increase. Randomness used to be synonymous with timeline of extreme infrequency. However, as systems distance themselves more and more from the Health Territory and deeper into Chaos, the random events get compressed into shorter and shorter time intervals. For example: during years 2012–2013, all within a span of several months, US experienced three colliding storms over North-East, estimated to be once in 100 year event and it produced hurricane Sandy in November 2012; housing bubble was thought to be 1:10,000 year event; Pope resigned, first time in 600 years; an asteroid/meteorite hit Earth and injured over 100 people in Siberia; global temperature was the highest in 4000 years. If societal systems remain in the extreme stage and accept it as a “new normal,” the ultimate consequences face the following scenario: either the horizontal hierarchy/people in the trenches attempt to control the system (a form of control through revolution) or the vertical/governing hierarchy attempts to control the system, analogous to a dictatorship.

Organized complexity is a hallmark of healthy clustered systems because it is capable of generating collective intelligence. This is contrary to disorganized complexity which is subject to random and reckless, non-system-optimizing crowed behavior with lack of collective intelligence, rationality, and responsibility (Wade, 2010; Collins, 2013).

Some chaos-associated diseases have already been observed to cluster. Serious mental illness, though a non-uniform group, places an individual bodily system in chaos; severe depression, however, is a reflection of entropy. Patients, grouped into “serious mental illness,” have been reported to be 2.6 times more likely to develop cancer than the general population (McGinty et al., 2012).

Acute infections are also chaos-related; they have been correlated with increased metastasis to the lung after acute bacterial infection (Smith and Kang, 2013).

As cancer cells rapidly multiply without differentiation in Chaos, they also rapidly age (Horvath, 2013; Mascarelli, 2013).

System's state, outside of Health Territory, affects its networks, including the metabolome, which impacts neuro-net. In vitamin A deficiency, a shortage in GABAergic neurons has been observed and such neurons are associated with Huntington's disease, autism, schizophrenia, and epilepsy (Chatzi et al., 2011). Similarly, vitamin D lack has been found and correlated with the severity of Parkinson's disease (Ding et al., 2013).

Mega-data expansion is analogous to unrestrained malignant biologic growth which allows a system to generate data without concomitant differentiation, e.g., gaining knowledge. Vision is a good example how to handle potentially massive input: it starts with a selective input followed by meaningful data filtration and compression, which is then presented to cognition for creation of information and knowledge. Hills and colleagues observed that “the more choices people have, the riskier the decisions they make” (Hills et al., 2013).

When the richness of input into a system's network begins to fade, there is regression of inter-connectedness; system enters entropy. Resiliency of a system comes from redundancy of network flow, its sources, diversity, gradient, velocity, etc. For example, it has been documented that bilingual patients developed dementia several years later than the monolingual ones (Alladi et al., 2013; Editorial, 2013).

Societies may express features of entropy, symptoms of degeneration. Neil Ferguson highlighted some *key features*; systems science equivalents are listed here in []: *Breakdown of the contract between generations* [trans-generational relationships are failing]; *Excess regulation* [dominance of vertical hierarchy]; *Decline of civil society* [lack of trust]; *Regulatory Excess* [disorganized complexity]; *Dependency on government to solve social issues* [giving up self-organization in favor of dependency on vertical hierarchy destabilizes system] (Ferguson, 2013).

In entropy, there is an increase of non-functionality due to the interruption of relationships via synaptic activity that lacks the balance between excitatory and inhibitory neurotransmitters, favoring inhibition. Both Alzheimer's and Parkinson's diseases are considered to be synaptopathies. Rise of psychiatric illnesses in a society is a sign of non-optimal network relationships (Barnes and Yaffe, 2011; Schipanski et al., 2013).

Most networks of biologic systems are an expression of temporary relationships. Exercise develops and maintains the density of neuro-muscular junctions, the connectome, which shows various ratios of muscle fibers per neuro-muscular junction. Lack of gradient flow, found in entropy, results in devolution of post-synaptic receptors. Once they are lost, it usually is permanent. The disorganized complexity of entropy in neuro-degenerative diseases manifests vanishing synaptic connections, both within brain and between the brain and the muscles; first clinical manifestations may show dysfunction of fine muscles, those with the highest density of neuromuscular junctions per bundle of muscle fibers, like the vocalis and intrinsic muscles of the hand, give us observable patients' difficulties in singing (especially hitting high notes) or failing handwriting; full loss of muscular strength, speed and coordination of walking follow, and herald dominating entropy (Funk et al., 2011; Rosenblum et al., 2013).

Some diseases, characterized for their occurrence in entropy, e.g., degeneration, may lessen the possibility of developing another disease associated with chaos, such as cancer. For example, neurodegenerative diseases, such as Parkinson's or Alzheimer's, are diseases of Entropy, but have been observed to have significantly below-average rate of cancer incidence, a disease of Chaos; the opposite exists as well, presence of cancer lessenes the chances for neuro-degeneration (Plun-Favreau et al., 2010; Musicco et al., 2013).

Attractors, (people, places, events, ideas, incentives, etc.), compete for dominance of awareness within system's neuro-net, while, correspondingly, suppressing existing ones; the stronger the attractor and its dominance, the less of cognition is available for other decisions needed for managing *change*; in most instances, however, there is an option to choose among attractors; multi-tasking may produce counter-currents. Goleman quotes Herbert Simon, recipient of 1978 Nobel in Economics: “A wealth of information creates a poverty of attention” (Goleman, 2013).

*Change* reflects materialization of new attractors which alter the existing flow through neuro-net; any leading awareness begins to restructure system's neuro-net which has the capacity to modify the epigenome (LeDoux, 2003). Once perceived, *change* alters the transient status quo of system's networks; perception indicates activation of senses and, simultaneously, sense-specific filtration and compression of incoming *change* which may, as a new system attractor, exert dominance over existing awareness within the neuro-net (Figures 2A–E).

The theoretical limit, of what can be quantified as risk by our senses, is determined by the range of capacity for sensory activation which is extremely limited. A useful metaphor follows: “if the entire spectrum of light is considered a distance from New York to Los Angeles, the spectrum, visible to us, is a dime”(NOVA, 2013).

Enhancement of our sensory perception with technology has a great potential to obtain further input from what was previously hidden from us, while respecting any inherent limitations in the instruments and the potential for misapplication by the operator. C*hange* then assumes a richer context of probability risk with less of uncertainty. Simultaneously, our cognitive paradigm and conscientious effort, however, need to keep pace in order to be capable of creating ever-higher level of knowledge; otherwise, the non-optimizing stress of cognitive dissonance is likely to increase (Brody, 2013).

The study of vision shows the gaps among the vast information potential available in the spectrum of light and what actually activates the retina followed by engagement of the cognitive domain. Most of the information that we perceive does come from our vision, about 80%, with the remaining 20% supplied by our hearing and other senses. Nolte points out that “we are capable of perceiving light only in the visible range of the electromagnetic spectrum that excite the retina in human eyes and vary from about 0.4 microns (for violet color) to 0.7 microns (for red); retina itself has only a limited number of sensors and nerve endings that can be activated: retina contains about 120 million rods and about 6 million cones, but only about 1 million ganglion cells… [which means that] the light information falling on 126 photoreceptors produces only a single signal in one ganglion cell axon… the information convergence transforms the signals from 126 million receptors into only 1 million axons in the optic nerve… a spoken language proceeds at approximately 25 bits per second… [and] data rate for non-verbal information is virtually the same as the 25-bit-per-second rate for language comprehension” (Nolte, 2001; Huth et al., 2012).

Lifestyle choices do impact the neuro-net. For example, alcohol affects connectivity between the amygdale and the prefrontal cortex (Gorka et al., 2013).

Diminishing sensory input translates into correspondingly diminishing neuro-net. Important observation by researchers includes the correlation between hearing loss and dementia (Lin et al., 2013), between visual contrast sensitivity and physical functioning (Swindell et al., 2010) and diminished olfaction in early stages of degenerating neuro-net (Doty, 2013).

There are gender differences in neuro-net wiring with greater neural connectivity from front to back and within one hemisphere in males and between the left and right hemispheres in females (Ingalhalikar et al., 2013).

*Changes* in neuro-net are usually followed by a degree of *change* in its system's epigenome ending as *changes* in the morphology of the system's phenotype. A neuro-net, which is sustaining a dominant awareness, expressed in parallel decisions and effort can create an epigenome reflective of the induced *changes*; it can happen within a few milliseconds to decades.

The consequence of decisions-altered epigenome may vary greatly; while it takes only about 300 milliseconds for our decision to bring an arm with a cigarette to the mouth, it may take 20+ years to develop lung cancer; a similar path exists for obesity, degenerative diseases, etc. (Nolte, 2001; Churchland et al., 2012; Frost, 2013; Horvath, 2013).

The mosaic of any epigenome reflects the UP/DOWN activation of genes through many life choices; it is shared by forebears with offsprings in a trans-generational impact; it reflects activation/deactivation of genes in response to induced *change*. Systems science indicates that, for example, generations of non-optimized systems (parents/grandparents, etc.,), which produced non-optimized outputs in response to *change* they faced, transferred their mis-activated/non-optimized genes to the subsequent generations. The morphologic development of a new offspring, in its first Life Phase (25± years), the Ancestral Phase, is strongly controlled by genes that were activated/de-activated by our parents/grandparents, etc.; having a baby in teen years has a high potential for transmitting the same mis-activated genes to the next generation without the opportunity to modify them during the subsequent Decision Life Phase. In addition, if, during this second Life Phase, the next 25± years, the choices that a young adult makes in response to *change* are further non-optimizing, it causes additional epigenetic mis-activation, perpetuating, or worsening disorganized complexity with corresponding epigenetic modifications (American Public Health Association, 2012; Linschooten et al., 2013; Oury et al., 2013; Padmanabhan et al., 2013; Pera, 2013; Ridaura et al., 2013).

Relationships are directly linked to system's capacity to respond to *change* as well as what *change* it generates.

Relationships principles that sustain a healthy biologic system, such as reciprocity, fairness, empathy, and trust with gratitude are considered to represent the foundation of morality (deWall et al., 2009). Gratitude reflects the focus on the positives (Seligman, 2012).

Relationships, with their feedback loops, are central to the function and structure of a biologic system, its clusters and inter-related systems, what type of *change* it generates and how competently it responds to ones that it receives (Cross, 2010). Relationships are based on flow of energy/information. The relationships among sub-systems, and their contributions to the larger system's emergence/output, are variable and not always harmonious; some function in Health Territory, while others may be in Chaos or Entropy, giving rise to a system-wide stressful dissonance.

Loss of trust leads to loss of common sense that precipitates loss of confidence because the foundation for rationally judging the world, making decisions, etc. disappears. Without prevailing societal trust, any *change,* distributed within socio-economic system, will have a strong tendency to spiral into ill-defined uncertainty. Only truth leads to trust and without trust there is no optimizing relationship; in its absence, there is no organized complexity to create value and randomness takes a center stage (van Gigch, 2007; Friedman, 2009). In 2013, even the Nobel Committee was not sure which observation of *change,* in the sphere of economics, was more plausible and thus to receive their full trust: Fama's theory that asset prices perfectly reflect all available information or Shiller's evidence of irrational, inefficient behavior? (Appelbaum, 2013).

### Flow through networks propagates change

The flow of information originates with sensory perception; its processing is subject to cognitive filters of assessor's hermeneutics; it is the flow of energy and information that sustains networks. Relationships, which exchange energy/information, may also be referred to, by Quantum Physics' term “entanglements,” which linguistically captures to complexities of network feedback loops. Relationships are temporary, unstable, and relative to the stratification within a pertinent system cluster which reflects its culture and the relative standing vis-à-vis other members. Flow is influenced by attractors; health territory has mostly complementary attractors; entropy has absence of attractors and chaos has a few super-dominant attractors.

Sleep is a key biologic cycle (Pack, 2009; Yu et al., 2013). Healthy flow through a system is never constant and the progressions/regressions form cycles. The most critical biologic cycle is the circadian rhythm which receives the signals for its resetting via light and darkness. Sunlight entrains the circadian cycle; as a consequence, the metabolic cycles, generating reactive oxygen species, are responsible for the level of oxidative stress and its impact on cognition (Rey and Reddy, 2013).

What is emerging from experimental evidence is that sleep is essential for the maintenance of the neuro-net (Xie et al., 2013).

The night portion of daily circadian rhythm represents the re-setting of each individual biologic system with up-regulation of SIRT-1 system-optimizing genes, associated with healthy longevity. Without the rhythmicity of day/night oscillations, biologic systems, as studied in laboratory animals, tend to falter, live shorter life spans and develop various degenerative/entropy-characteristic diseases.

Network flow is, to a large extent, proportionate to education, either self-generated or obtained through an organized process; various societal studies strongly parallel achievements with education (Lopatto, 2012).

Output, system's emergence, is a direct consequence of *changes* within a system, either self-generated or externally induced.

Cognition is the emergence of a synaptic network; “every time we learn something we change the brain to help us learn something else” (LeDoux, 2003).

The processing of any received data/information via senses goes through the paradigm of an assessor which should be based on current-science-based rationality as a background for experiential confidence. For example, as a measure of likely “mastery” of a subject and to be considered an “expert,” the rule of “10 years/10,000 hours” reflects the need for sustained and prolonged dominance of cognitive awareness/learning with focus on specific skill which is being accompanied by conscientious effort (Chase and Simon, 1973; Syed, 2010).

Paradigm is the reality that each of us lives in, how we think that we know and understand what is happening; it forms the basis for our decisions. “Behavioral economics [explores] how people misinterpret information, how their emotions distort their decisions, and how they miscalculate probabilities” (Mandelbrot, 2004).

Your paradigm determines your hermeneutics, your world view determines your method of interpretation. The paradigm that we use filters/affects what we perceive/see and hear (Berger and Ehrsson, 2013).

During the lifetime of a biologic system, neuro-net is undergoing unending construction and destruction, repair and neglect, all reflected in cognition. *Change* may trigger sensory activation. Senses in conjunction with cognition, which is variable and conditional, can determine the fluctuating proportions of the risk/uncertainty ration and its interpretation. The R/U ration, proportionately to the size of the denominator, reveals the level of remaining uncertainty and with it, the emerging stress as an expression of cognitive dissonance (Festinger, 1957). Cognitive dissonance creates stress that epigenetically negatively impacts the methylome (Junger and van Kampen, 2010; Puterman et al., 2010). Persistent dominance of awareness, by non-optimizing attractors, likely leads to chronic stress (Blackburn and Epel, 2012; Nester, 2012).

The recorded data of the financial markets reflect human decisions. The Kondratieff's Long Wave, charting *changes* in price/credit of commodities, can serve as a general proxy for the level of prevailing trust within the societal system's inter-relationships. Ascend to top of Long Wave, estimated to have been reached around the year 2000, paralleled dilution of trust and loss of relationships during the preceding years. In 1985, for example, “*most people said they had three close friends; in 2004 the most common number was zero*” (Lieberman, 2013).

*Change* as a system's emergence/output, can be either positive or negative; it arises at multiple crossroads of networks relationships. Emergence/output can amount to value, categorized here as a composite of efficiency, effectiveness, risk management, and proportionate cost in processed energy and information; the opposite, a non-value output lacks such features; a system that generates value is also referred to as a complex adaptive system that is capable of successful adapting and evolving with *change*.

This research represents personal understanding of systems science derived from hands-on engagement with human health and illness, observations of biology as well as perspectives derived from other researchers, business, and management fields. The extracts, included in the Materials section, offer reader an avenue for corroboration of results derived from this research, or their modification, as any observed event or reported finding may have different meaning for different observers; if that is the case with this study—readers' exploration of data, information, knowledge reported in the text—it would support the validity of this contribution. It is hoped that this study will provide a stimulus for further discussion and study, as *change* of biologic systems never ceases and our knowledge will always be a step behind.

## Conclusions

Life of biologic systems is an endless *change*, ever evolving or devolving, with inseparable and complementary process and outcome, two theaters but in one larger whole. The process is centered on flow of energy and information through networks of relationships, and the outcome becomes the consequence.

*Change* is never an isolated event; its understanding requires context; it is also not homogeneous but is composed of innumerable *changes* arising from other systems. Systems science offers a unique perspective for integrating *change* into a multidimensional context and the extraction of knowledge. It provides tools to examine and react to *change* pragmatically with guarded optimism based on a favorable risk/uncertainty ration.

*Change* represents altered relationships and ends by altering others; it is observed on any and all levels studied by science, from cellular to societal systems. Biologic entities are capable of registering a portion of *change* within the boundaries of their senses; what is recorded may be considered a risk-probability; what is outside the sensory range is an uncertain possibility. *Change* is seen as an inseparable composite of risk and uncertainty but in variable ratios, influenced by sensory perception and judgment.

Relationships of biologic systems are reflections of flow of energy and information through their networks and form the foundation of systems functional complexity which creates their output/emergence. Relationships that engage in reciprocity, fairness, empathy, and are based on trust, generate organized complexity with propensity to create value, conceptualized as efficiency, effectiveness, risk/*change* management, and proportionate cost.

The knowledge of systems science allows a prospective evaluation of *change;* it examines *change* in the light of system's optimizing or non-optimizing influence before it impacts other networks including the epigenome of self and others. Differentiating *change* into risk and uncertainty puts an identifiable boundary around sensory-derived probability of risk which diminishes the nebulous possibilities of uncertainty.

Attractors, which are visualized as guiding network flow, can be represented by people, places, events, ideas but also by diet, exercise, stress, simply by anything that achieves dominance over cognition; it affects decisions and effort. In turn, attractors-awareness-decisions-effort mosaic *changes* inter-related networks all the way to the genes. Epigenome is evolving with Life; it is *changing* from minutes to decades, in a single bodily system and through multiple generations; it impacts any related morphogenic phenotype and its state of health. Senses are the gateways of systems for data/information; microbiome with metabolome represent the entry for targeted energy.

How forebears handled *change* is likely imprinted in the epigenome that is inherited by the offspring, a trans-generational influence; this epigenome remains dominant during the first Ancestral Life Phase; subsequent epigenomic expressions, however, vary and are based primarily on choices made during the second, labeled Decisions Life Phase; in the third and final life phase, the Phase of Consequences, the epigenome expressions are mostly according to the pre-settings that took place in the preceding Decisions Life Phase; it is measurable in altered DNA methylation; the cycle continues forward.

Synaptogenesis, the foundation process of neuro-net, is developing primarily during embryogenesis and young adulthood while gradually diminishing through subsequent life phases; it reflects the type of flow of energy/information strongly influenced by major decisions of parents and the adult offsprings.

Synapses have the ability to learn and unlearn with *change*; strong attractors alter the flow patterns through the network creating preferences that cascade down to the epigenome; synapses need ongoing formation and pruning to be available for the next experience. Diminished sensory input handicaps the capacity of neuro-net to respond to *change* with adaptation and evolution.

Biologic systems reflect memories and awareness which are being processed by cognition, fully dependent on synaptic connections. These relationships/links are temporary and quite unstable as they rely on ongoing inflow-outflow of energy/information. The preservation of functional and structural integrity of neuro-net is essential to system's health.

*Change*-activated neuro-net likely differs with gender, opening the possibility of dissimilar cognitive response among men and women.

Dynamic Systems Model defines system's functional or dysfunctional states, a Health Territory and two outlier states, one Chaos and the other Entropy. Only a healthy system is capable of generating optimizing *change* and has the resiliency to adapt and evolve with incoming *change*.

The level of existing trust is the deterministic feature of relationships but is difficult to measure; the Kondratieff's Long Wave can serve as a general proxy. Though, originally conceptualized to reflect the fluctuating prices/credit of commodities, its inverse pattern does reflect the prevailing level of societal trust; credit and trust must be in balance; unrestrained credit/debt dilutes trust.

The key to any system's health thus lies in its relationships; if capable of generating organized complexity, relationships produces value; reigning supreme, in humans, it seems to be the relationship between the hippocampus/amygdale and the pre-frontal cortex; it affects cognition that has the capacity to alter inter- and intra-cellular relationships autonomically by expressing our decisions/behavioral/lifestyle choices through impacting UP/DOWN regulation of our genes. The outcome, from thoughts/decisions to morphology, seems to be a highly dependent cascade.

### Going forward—pragmatic guidelines from systems science

To distinguish an optimized system from a non-optimized one—look at its complexity and examine the historic output/emergence; was there value creation?

Rebalance relationships to be reciprocal, fair, empathic, and based on trust; construct organized complexity; insist on value.

Convert uncertainty to risk whenever possible utilizing sensory input; learn how your team-mates asses *change*.

Know your attractors and protect your awareness as both represent gateways to your system's networks and cognition.

Understand the larger-systems' trends as well as biologic cycles; asynchrony often leads to cognitive dissonance.

### Conflict of interest statement

The author declares that the research was conducted in the absence of any commercial or financial relationships that could be construed as a potential conflict of interest.
